RETRACTED

# LIFR-AS1 modulates Sufu to inhibit cell proliferation and migration by miR-197-3p in breast cancer

**DOI:** 10.1042/BSR20180551

**Published:** 2019-07-08

**Authors:** Fangfang Xu, Hui Li, Chengjiu Hu

**Affiliations:** 1 Department of Pathology, Jining No.1 People’s Hospital, Jining 272011, China; 2 Department of Oncology, Affiliated Hospital of Jining Medical University, Jining 272100, China

**Keywords:** breast cancer, cell migration, miR-197-3p, LIFR-AS1, Sufu

## Abstract

Numerous evidence has recently demonstrated that long non-coding RNAs (lncRNAs) play vital roles in the oncogenesis and development of a wide range of human neoplasms. Leukemia inhibitory factor receptor antisense RNA 1 (LIFR-AS1), a novel cancer-related lncRNA, has been reported to be under-expressed in breast cancer and associated with poor prognosis. However, the exact role of LIFR-AS1 in breast cancer remains largely unclear. The present study aimed to investigate the biological role of LIFR-AS1 in breast cancer and clarify the potential molecular mechanisms. In the present study, we found that LIFR-AS1 was significantly down-regulated in both tissues and cell lines. Furthermore, over-expression of LIFR-AS1 inhibited breast cancer cell proliferation, colony formation, migration and invasion, whereas knockdown of LIFR-AS1 promoted breast cancer cell proliferation, colony formation, migration and invasion. Moreover, LIFR-AS1 was observed to up-regulate suppressor of fused gene (*Sufu*) expression by competitively binding to miR-197-3p in breast cancer cells. Notably, miR-197-3p inhibitor reversed the promoting effects of LIFR-AS1 knockdown on breast cancer cell proliferation, colony formation, migration and invasion. Additionally, LIFR-AS1 knockdown promoted tumor growth *in vivo*. To sum up, our results imply the tumor-suppressing role of LIFR-AS1 in breast cancer.

## Introduction

Breast cancer is one of the most common causes of cancer-associated mortality among the women worldwide [1,2]. It is estimated that over 1 million new breast cancer cases are diagnosed and roughly 370000 patients die of breast cancer around the world annually [3,4]. In the United States, 228000 new breast cancer cases and 40000 breast cancer-related deaths were estimated to occur every year [5,6]. Distant metastasis and drug resistance may account for the majority of breast cancer-related deaths [7,8]. In spite of recent advances in the diagnosis and therapy of breast cancer, the long-term survival is still unfavorable. Therefore, there is an urgent need to identify sensitive prognostic biomarkers and develop effective therapeutic strategies for breast cancer.

Long non-coding RNAs (lncRNAs) are a large class of non-protein-coding RNA transcripts larger than 200 nucleotides in length, which possess diverse biological functions [9,10]. Increasing studies have demonstrated that the ectopic expression of lncRNAs is implicated in various types of human disorders [11–13]. Evidence is accumulating that lncRNAs may serve as an miRNA sponge to exert their roles in the carcinogenesis and progression of human cancers [14,15]. Leukemia inhibitory factor receptor antisense RNA 1 (LIFR-AS1), a novel cancer-related lncRNA, is transcribed from the *LIFR* gene located on human chromosome 5p13.1 in an antisense manner [16]. A previous study has reported that LIFR-AS1 is under-expressed in breast cancer and associated with poor survival of breast cancer patients [17]. However, the exact role of LIFR-AS1 in breast cancer and its potential molecular mechanisms remain largely unknown.

RETRACTED

It is well documented that suppressor of fused (Sufu) is a negative regulator of Hedgehog signaling cascade, and represses the expression of the glioma-associated oncogene homolog (Gli), a Hedgehog signaling pathway downstream effector [18,19]. Hedgehog signaling pathway plays critical roles in a variety of cellular processes, such as cell proliferation, cell differentiation and cell fate determination [20,21]. Previous studies have demonstrated that Sufu acts as a tumor suppressor in several types of human tumors [22–24].

The present study aimed to explore the biological role of LIFR-AS1 in breast cancer and elucidate the potential molecular mechanisms involved. In the present study, we found that LIFR-AS1 was significantly down-regulated in both breast cancer tissues and cell lines. Functional investigations demonstrated that LIFR-AS1 exerted inhibitory effects on breast cancer cell proliferation, colony formation, migration and invasion. Moreover, mechanistic investigations revealed that LIFR-AS1 inhibits cell proliferation and migration via miR-197/Sufu axis in breast cancer.

## Materials and methods

### Patients and tissues specimens

Tumorous tissues and corresponding adjacent tissues were obtained from 30 patients in Jining No.1 People’s Hospital (Jining, China) from April 2014 to August 2016. Corresponding adjacent normal tissues were obtained at a distance of 5 cm from breast cancer tissues. All clinical samples were immediately frozen in liquid nitrogen and stored at −80°C for further experiments. The present study was supported by the Ethics and Scientific Committee of Jining No.1 People’s Hospital. All the patients enrolled in the present study gave written informed consent.

### Cell culture

A normal human breast epithelial cell line Hs 578Bst and four breast cancer cell lines (MDA-MB-415, MDA-MB-231, MDA-MB-468 and MCF7) were purchased from Shanghai Cell Bank, Chinese Academy of Sciences (Shanghai, China). All the cells were cultured in DMEM (Gibco, Grand Island, New York, U.S.A.) supplemented with 10% fetal bovine serum (FBS, Sigma–Aldrich, St. Louis, MO, U.S.A.). Cells were maintained at 37°C in a humidified atmosphere containing 5% CO_2_.

RETRACTED

### Cell transfection

Cell transfection was carried out using Lipofectamine 2000 (Invitrogen, Waltham, U.S.A.) according to manufacturer’s instructions. Cells (5 × 10^5^ cells per well) were transfected with LIFR-AS1 or si-LIFR-AS1. LIFR-AS1 mimics and small interfering RNA to knockdown LIFR-AS1 were synthesized by Shanghai GenePharma Co., Ltd. (Shanghai, China). Cells were harvested 48 h post-transfection for further studies.

### RNA isolation and quantitative real-time polymerase chain reaction

Total RNA and microRNAs were extracted from tissues and cells using TRIzol reagent (Qiagen, Hilden, Germany) according to the manufacturer’s protocol. Following quantitation by Nanodrop 2000 (Thermo Fisher Scientific, Waltham, U.S.A.), the extracted total RNA was reverse-transcribed using Reverse Transcription Kit (Takara, Dalian, China). RT-PCR was performed on an Applied Biosystems 7500 Fast Real-Time PCR systems (Applied Biosystems). The specific primer sequences were synthesized by Shanghai Sangon Biological Engineering Technology and Service. The PCR conditions were as follows: denaturation at 95°C for 10 min, followed by 40 cycles of 95°C for 5 s and 60°C for 40 s. β-actin was used as an endogenous control to normalize LIFR-AS1 and Sufu expression levels. The relative expression level was calculated using the 2^−ΔΔ*C*^_t_ method. The experiments were performed in triplicate.

### *In situ* hybridization

Tissue slides were pre-hybridized in a hybridization solution (Boster Bioengineering Co., Ltd, Wuhan, China) at 37°C for 2 h. Ten picomoles of digoxigenin-labeled detection probes (Boster) complementary to LINC00461 were added and hybridized overnight at 37°C. After stringent washes, an immunologic reaction was carried out using a mouse monoclonal antibody to digoxigenin (ab6212), followed by adding alkaline phosphatase–conjugated streptavidin dilution (BD Bioscience) to detect streptavidin dilution probes. Slides were mounted with aqueous mounting medium (Maixin Biotechnology, Fuzhou, China).

### Cell proliferation

Cells were seeded at the concentration of 5 × 10^3^ cells/well in 96-well plates at 24 h after transfection. Cell proliferation was measured using MTT Cell Proliferation and Cytotoxicity Assay Kit (Sigma–Aldrich, St. Louis, U.S.A.). Following incubation at 37°C for different periods of time (0, 24, 48 and 72 h), the culture medium was removed and MTT (20 μl; 5 mg/ml) was added to each well. After incubation at 37°C for another 4 h, MTT solution was removed and replaced with dimethyl sulfoxide (DMSO; 150 μl, 4%; Sigma–Aldrich). Absorbance was determined at 560 nm after using a microplate spectrophotometer (Thermo Labsystems, Vantaa, Finland).

RETRACTED

### Colony formation analysis

Cells were trypsinized, counted and seeded into 12-well plates at the concentration of 100 cells per well. The medium was replaced every 3 days during the colony growth. After incubation in DMEM for 12 days, the colonies were fixed with methanol and stained with Crystal Violet (Sigma–Aldrich, U.S.A.). The colonies were counted under an inverted microscope (Nikon, Japan).

### Wound healing assays

Cells were seeded in six-well culture plates to grow into a monolayer (basically 100% confluence). The cell monolayer was scraped using pipette and washed twice with medium to form a wound. The cells were further cultured in the medium for 24 h and closure of scratch was observed using an inverted microscope (Olympus). Cells were observed at 0 and 24 h after scraping under an inverted microscope and corresponding photographs were taken. The cell-free area at 24 h after wounding and original denuded area were measured using the ImageJ software (National Institutes of Health, Bethesda, MD, U.S.A.).

### Transwell invasion assay

Transwell invasion assay was performed to evaluate cell invasion. The upper surface of the a filter (pore size, 8.0 μm; Biosciences, Heidelberg, Germany) was coated with basement membrane Matrigel (BD Bioscience), at a concentration of 2 mg/ml and incubated at 4°C for 3 h. A total of 2 × 10^4^ cells were seeded into upper chamber with 200 μl serum-free medium. The lower chamber was supplemented with 750 μl medium containing 10% FBS. Following incubation for 24 h at 37°C, cells were fixed with 4% polyoxymethylene and stained with 0.5% Crystal Violet (Sigma–Aldrich). Then stained cells were observed and counted under a microscope. Five visual fields were selected and the average number was taken.

### RNA-binding protein immunoprecipitation

RNA-binding protein immunoprecipitation (RIP) assays were carried out using EZ-Magna RIP™ RNA-Binding Protein Immunoprecipitation Kit (Millipore, Billerica, MA, U.S.A.) in accordance with manufacturer’s instructions. Briefly, RIP buffer containing magnetic beads conjugated with human anti-Ago2 antibody (Millipore) or negative control IgG (Millipore) was added to cell lysate, and subsequently incubated for overnight at 4°C. Proteinase K was applied to digest the proteins and then the co-precipitated RNAs were isolated. The purified RNAs were subject to RT-PCR analysis.

RETRACTED

### Xenograft tumor model assay

All animal experiments were performed in accordance with institutional and international animal regulations. Animal protocol was approved by Jining No.1 People’s Hospital. Female BALB/c nude mice (6 weeks of age) were purchased from Beijing HFK Bioscience Co., Ltd. (Beijing, China). MDA-MB-415 cells transfected with sh-NC or sh-LIFR-AS1 (1 × 10^6^ cells per mouse) were subcutaneously administrated into the flanks of BALB/c nude mice, respectively. The length and width of tumors were measured using a caliper every 5 days. All mice were killed at day 35 post-injection, and the tumor nodules of the mice were removed and weighed. The tumor volume was calculated according to the following equation:

$$\text{tumor volume }({\text{mm}}^{3})\;=\;\text{length }(\text{mm})\;\times \;{\text{width (mm)}}^{2}/2.$$

### Immunohistochemistry assay

Samples were fixed in 10% neutral buffered formalin, embedded in paraffin, and sliced into thin sections (5 μm). After being dewaxed and rehydrated, sections were incubated with 3% H_2_O_2_ for 30 min to block the endogenous peroxidase (POD) activity. Following antigen retrieval (AR) by microwave (heating), 5% bovine serum albumin (BSA) was applied to block nonspecific binding. The sections were then incubated with primary antibodies at 4°C overnight. Anti-Ki67 (ab15580) and anti-Sufu (ab28083) were obtained from Abcam (Cambridge, MA, U.S.A.) and used at a dilution of 1:200. After being rinsed with phosphate-buffered saline (PBS) three times for 5 min each, sections were treated with biotinylated secondary antibody (Abcam, Cambridge, U.S.A.) for 1 h, followed by incubation with streptavidin-horseradish peroxidase (HRP) for 20 min. Diaminobenzidine (DAB) substrate was used as the color developing agent for visualization of Ki67-positive cells.

### Western blotting analysis

Protein lysates were extracted from cells using 500 μl radio immunoprecipitation assay (RIPA) buffer with 1 mM phenylmethane sulfonyl fluoride. Samples were subsequently sonicated for 2 min and centrifuged. The supernatants were collected and used for protein analysis. Lysates were separated on 8% polyacrylamide gels and transferred on to PVDF membrane. The membranes were blocked with PBS containing 0.1% Tween-20 (PBST) and 5% nonfat milk (w/v) for 1 h at room temperature. After they were washed with PBST, the membranes were probed with antibodies overnight at 4°C. Primary antibodies were purchased from Abcam and used at the following dilutions: anti-Sufu (ab28083, 1:500) and anti-β-actin (ab6276, 1:1000). The membranes were washed again with PBST, then HRP-labeled IgG at 1:5000 dilution was added at room temperature for 1 h, and the blots were developed using ECL Western blotting reagents.

RETRACTED

### Luciferase reporter assay

Wild-type Sufu 3′UTR fragment and mutant Sufu 3′UTR fragments were inserted into pmirGLO reporter vectors (Promega, Madison, WI, U.S.A.), respectively. Cells were co-transfected with miR-197-3p mimics and wild-type Sufu 3′UTR or mutant Sufu 3′UTR fragments by Lipofectamine 2000 (Invitrogen). Relative luciferase activity was measured on a dual-luciferase reporter assay system (Promega) at 48 h post-transfection. Data were expressed as the ratio of *Renilla* luciferase activity to firefly luciferase activity.

### Statistical analysis

Data were expressed as mean ± standard deviation (SD). Statistical analysis was carried out using SPSS 16.0 software (SPSS, Chicago, IL, U.S.A.). Two-tailed Student’s *t* test was employed to compare the differences between two groups and one-way analysis of variance (ANOVA) followed by Dunnett’s multiple comparison was applied to compare the differences among three independent groups. *P*<0.05 was considered statistically significant.

## Results

### LIFR-AS1 is significantly down-regulated in breast cancer tissues and cell lines

LIFR-AS1 has been reported to be under-expressed in breast cancer and associated with poor survival, however its exact role in breast cancer remains largely unknown. To investigate the biological role of LIFR-AS1 in breast cancer, we initially analyzed LIFR-AS1 expression data downloaded from TCGA database and found that LIFR-AS1 was significantly down-regulated in cancerous tissues compared with normal breast tissues (Figure 1A). We subsequently conducted quantitative real-time polymerase chain reaction (qRT-PCR) and ISH analyses to determine the expression of LIFR-AS1 in tumorous tissues and matched non-cancerous tissues. In agreement with TCGA data, cancerous tissues showed lower LIFR-AS1 expression levels than corresponding adjacent non-tumorous tissues (Figure 1B,C). Consistently, LIFR-AS1 was found to be markedly down-regulated in breast cancer cell lines compared with normal human mammary epithelial cell line Hs 578Bst (Figure 1D). Our results suggest that LIFR-AS1 is significantly down-regulated in both breast cancer tissues and cell lines.

**Figure 1:** LIFR-AS1 is significantly down-regulated in breast cancer tissues and cell lines (**A**) LIFR-AS1 expression data in breast cancer tissues and normal tissues were downloaded from the TCGA database. (**B**) LIFR-AS1 expression levels in 30 pairs of breast cancer tissues and matched paracancerous tissues were determined by qRT-PCR. (**C**) LIFR-AS1 expression in breast cancer tissues and adjacent normal tissues was visualized by ISH. (**D**) The expression levels of LIFR-AS1 in one normal human epithelial cell line Hs578Bst and four breast cancer cell lines (MDA-MB-415, MDA-MB-231, MDA-MB-468 and MCF7) were determined by qRT-PCR. **P<0.01, ***P<0.001.

RETRACTED

### LIFR-AS1 inhibits breast cancer cell proliferation and colony formation

To investigate the biological role of LIFR-AS1 in breast cancer, we performed over-expression studies in MCF7 cells and knockdown studies in MDA-MB-415 cells, respectively. Transfection efficacy was identified using qRT-PCR analysis (Figure 2A). As presented in Figure 2B, LIFR-AS1 over-expression dramatically suppressed MCF7 cell proliferation compared with control group, whereas LIFR-AS1 down-regulation markedly expedited MDA-MB-415 cell proliferation. As evident from colony formation assays, LIFR-AS1 over-expression significantly repressed the clonogenic abilities of MCF7 cells in comparison with control treatment, while LIFR-AS1 down-regulation remarkably contributed to MDA-MB-415 cell proliferation (Figure 2C). Our data manifest that LIFR-AS1 suppresses breast cancer cell proliferation and colony formation.

**Figure 2:** LIFR-AS1 inhibits breast cancer cell proliferation and colony formation (**A**) LIFR-AS1 expression levels in breast cancer cells were determined by qRT-PCR after treatment with LIFR-AS1 mimics or siLIFR-AS1. (**B**) Breast cancer cell proliferation was examined by CCK8 assays after treatment with LIFR-AS1 mimics or siLIFR-AS1. (**C**) Colony formation assays were carried out to detect the clonogenic ability of breast cancer cells after treatment with LIFR-AS1 mimics or siLIFR-AS1. **P<0.01, ***P<0.001.

### LIFR-AS1 inhibits breast cancer cell migration and invasion

To explore whether LIFR-AS1 affects the motility of breast cancer cells, we assessed the migration and invasion abilities of breast cancer cells after treatment with LIFR-AS1 or si-LIFR-AS1. As evident from wound healing assays, LIFR-AS1 over-expression notably slowed down MCF7 cell migration compared with control group, whereas LIFR-AS1 down-regulation dramatically accelerated MDA-MB-415 cell migration (Figure 3A). As presented in Figure 3B, LIFR-AS1 over-expression significantly inhibited the invasion abilities of MCF7 cells compared with control treatment, while LIFR-AS1 knockdown dramatically strengthened the invasion capabilities of MDA-MB-415 cells. Our results indicate that LIFR-AS1 represses breast cancer cell migration and invasion.

**Figure 3:** LIFR-AS1 inhibits breast cancer cell migration and invasion (**A**) Breast cancer cell migration was analyzed by wound healing assays after treatment with LIFR-AS1 mimics or siLIFR-AS1. (**B**) Breast cancer cell invasion was analyzed by transwell invasion assays after treatment with LIFR-AS1 mimics or siLIFR-AS1. **P<0.01, ***P<0.001.

RETRACTED

### LIFR-AS1 interacts with miR-197-3p in breast cancer cells

Accumulating studies have demonstrated that lncRNAs serve as miRNA sponge to exert their functions in diverse types of human malignant neoplasms. To shed some light on the potential molecular mechanisms by which LIFR-AS1 inhibits breast cancer cell proliferation, migration and invasion, we performed bioinformatics analysis and applied miRanda online software to predict the potential targets of LIFR-AS1. MiR-197-3p, frequently reported to act as an oncogene in several types of human tumors, was selected as a candidate target of LIFR-AS1 (Figure 4A). To verify the interaction between miR-197-3p and LIFR-AS1, anti-Ago2 RIP assays were conducted. As obvious from Figure 4B, miR-197-3p was remarkably enriched by LIFR-AS1 over-expression treatment compared with control group. As presented in Figure 4C, MCF7 cells treated with LIFR-AS1 mimics exhibited lower miR-197-3p expression levels than control treatment, whereas higher miR-197-3p expression levels were observed in MDA-MB-415 cells transfected with si-LIFR-AS1. Our results suggest that LIFR-AS1 interacts with miR-197-3p in breast cancer cells.

**Figure 4:** LIFR-AS1 interacts with miR-197-3p in breast cancer cells (**A**) A putative binding site of miR-197-3p in LIFR-AS1 was predicted by miRanda algorithms. (**B**) Anti-Ago2 RIP was carried out to enrich the RNAs interacting with LIFR-AS1 in MCF7 cells after treatment with negative control or LIFR-AS1 mimics. (**C**) MiR-197-3p expression levels were determined by qRT-PCR after treatment with LIFR-AS1 mimics or siLIFR-AS1. ***P<0.001.

### LIFR-AS1 modulates Sufu expression by sponging miR-197-3p in breast cancer cells

Mounting studies have showed that lncRNAs may act as competing endogenous RNAs (ceRNAs) to sequester miRNAs from their corresponding target mRNAs. To further clarify the potential molecular mechanisms underlying breast cancer tumorigenesis and development, we applied miRanda algorithms to predict the possible targets of miR-197-3p. Among all the putative targets of miR-197-3p, Sufu drew our attention for its importance in the carcinogenesis and progression of diverse types of human cancers (Figure 5A). To verify the binding of miR-197-3p and Sufu, we conducted dual luciferase reporter assays. As presented in Figure 5B, co-transfection of miR-197-3p and wild-type Sufu 3′UTR fragment markedly decreased the luciferase activity, whereas co-transfection of miR-197-3p and mutant Sufu 3′UTR fragments failed to alter the luciferase activity. Furthermore, miR-197-3p mimics were noticed to inhibit Sufu protein expression compared with negative control group (Figure 5C). In addition, co-transfection of si-LIFR-AS1 and wild-type Sufu 3′UTR fragments was found to reduce the luciferase activity, while co-transfection of si-LIFR-AS1 and mutant Sufu 3′UTR fragments failed to change the luciferase activity (Figure 5D). Moreover, LIFR-AS1 knockdown was observed to repress Sufu protein expression compared with negative control treatment (Figure 5E). Our results suggest that LIFR-AS1 knockdown has similar effects on Sufu protein expression with miR-197-3p mimics. To sum up, LIFR-AS1 modulates Sufu expression by sponging miR-197-3p in breast cancer cells.

RETRACTED

**Figure 5:** LIFR-AS1 up-regulates Sufu expression in breast cancer cells by sponging miR-197-3p (**A**) A putative binding site of miR-197-3p in the 3′UTR of Sufu was predicted by miRanda algorithms. (**B**) Luciferase activity was examined after co-transfection of miR-197-3p and wild-type Sufu 3′UTR fragment or mutant Sufu 3′UTR fragment. (**C**) Sufu protein expression was examined by Western blotting after treatment with negative control or miR-197-3p mimics. (**D**) Luciferase activity was determined after co-transfection of siLIFR-AS1 and wild-type Sufu 3′UTR fragment or mutant Sufu 3′UTR fragment. (**E**) Sufu protein expression was examined after treatment with negative control siRNA or siLIFR-AS1. ***P<0.001.

### MiR-197-3p inhibitor reverses the promoting effects of LIFR-AS1 knockdown on breast cancer cells

As shown in Figure 6A,B, miR-197 mimics significantly facilitated breast cancer cell proliferation and invasion, whereas miR-197 inhibitor dramatically inhibited breast cancer cell proliferation and invasion. To explore whether the effects of LIFR-AS1 on breast cancer cells are mediated by miR-197-3p, we down-regulated the expression of miR-197-3p in breast cancer cells treated with si-LIFR-AS1. As shown in Figure 6C–F, miR-197-3p inhibitor reversed the promoting effects of LIFR-AS1 knockdown on breast cancer cell proliferation, colony formation, migration and invasion. In addition, miR-197-3p inhibitor was also found to reverse the inhibitory effects of LIFR-AS1 on Sufu protein expression (Figure 6G) Our data indicate that miR-197-3p mediates the effects of LIFR-AS1 on breast cancer cell proliferation, migration and invasion.

**Figure 6:** MiR-197-3p inhibitor reversed the promoting effects of LIFR-AS1 knockdown on breast cancer cells (**A**) Cell proliferation was determined by CCK8 assays after transfection with miR-197 mimics or miR-197 inhibitor. (**B**) Cell invasion was detected via Transwell invasion assays after transfection with miR-197 mimics or miR-197 inhibitor. (**C**) MDA-MB-415 cell proliferation was examined by CCK8 assays after co-transfection of miR-197-3p inhibitor and siLIFR-AS1. (**D**) Clonogenic ability of MDA-MB-415 cells were determined by colony formation assays after co-transfection of miR-197-3p inhibitor and siLIFR-AS1. (**E**) MDA-MB-415 cell migration was examined by wound healing assays after co-transfection of miR-197-3p inhibitor and siLIFR-AS. (**F**) MDA-MB-415 cell invasion was determined by transwell invasion assays after co-transfection of miR-197-3p inhibitor and siLIFR-AS1. (**G**) Sufu protein expression in MDA-MB-415 cells was detected by Western blot analysis after co-transfection of miR-197-3p inhibitor and siLIFR-AS1. **P<0.01, ***P<0.001.

RETRACTED

### LIFR-AS1 knockdown promotes tumor growth *in vivo*

Xenograft tumor model assays were conducted to evaluate the effect of LIFR-AS1 knockdown on tumor growth *in vivo*. As shown in Figure 7A, LIFR-AS1 knockdown dramatically suppressed growth *in vivo*. Moreover, IHC analysis demonstrated that LIFR-AS1 knockdown inhibited Ki67 expression in the collected tumors (Figure 7B). qRT-PCR analysis showed that LIFR-AS1 knockdown dramatically miR-197-3p expression in the collected tumors (Figure 7C). Furthermore, LIFR-AS1 knockdown was observed to repress Sufu protein expression in the tumors (Figure 7D). Our results suggest that LIFR-AS1 knockdown inhibits tumor growth *in vivo*.

**Figure 7:** LIFR-AS1 knockdown promoted tumor growth *in vivo* (**A**) MDA-MB-415 cells treated with negative control siRNA or siLIFR-AS1 were injected into the flanks of the nude mice (*n*=5). The tumor volumes were measured every 5 days using a slide caliper; mice were killed at day 35 post-implantation, and the tumors were peeled off and weighted. (**B**) Ki67 protein expression in the collected tumors was examined by IHC. (**C**) MiR-197-3p expression levels in the collected tumors were detected by qRT-PCR. (**D**) Sufu protein expression in the collected tumors was examined by IHC. ***P<0.001.

## Discussion

Breast cancer is one of the most frequent gynecological malignant neoplasms among the women worldwide [25]. The incidence of breast cancer is rapidly increasing and it has brought great economic pressures and high health risks to the women around the world [26]. Previous studies have reported that targeting steroid receptor and inhibiting tumor-related signaling transduction are considered as promising treatment choices for human malignancies [27–29]. In spite of great progress in the diagnosis and therapy, the long-term survival is still unsatisfactory. Numerous evidence has revealed that lncRNAs are important regulators in the tumorigenesis and progression of diverse types of human cancers [11–14]. Previous studies have demonstrated that LIFR exerts tumor-suppressing functions in hepatocellular carcinoma [30]. LIFR-AS1 has been reported to be under-expressed in breast cancer and associated with poor survival [17]. Nonetheless, the exact biological role of LIFR-AS1 in breast cancer and its potential molecular mechanisms remains largely understood. Hence, a better understanding of the biological role of LIFR-AS1 may be helpful to generate novel therapeutic alternatives for breast cancer.

RETRACTED

In the current study, we first analyzed LIFR-AS1 expression data downloaded from TCGA database and discovered that LIFR-AS1 was significantly down-regulated in tumorous tissues. Next, we carried out qRT-PCR and ISH analyses to determine LIFR-AS1 expression in the collected clinical samples, and found that LIFR-AS1 expression in cancerous tissues was lower than that in matched non-cancerous tissues. Consistently, LIFR-AS1 was under-expressed in breast cancer cells. To gain a better understanding of the biological role of LIFR-AS1 in breast cancer, functional investigations were carried out. Moreover, functional studies have illustrated that LIFR-AS1 exerts inhibitory effects on breast cancer cell proliferation, colony formation, migration and invasion. In addition, LIFR-AS1 knockdown was observed to inhibit tumor growth *in vivo*. Our findings indicates that LIFR-AS1 may function as a tumor suppressor in breast cancer.

Mounting studies have demonstrated that lncRNAs act as miRNA sponge to exert their roles in the oncogenesis and development of human tumors. Previous studies have reported that miR-197-3p exerts tumor-promoting functions in a variety of human malignancies, such as bladder cancer [31], lung adenocarcinoma [32], ovarian cancer [33], pancreatic cancer [34], and non-small cell lung cancer [35]. It is acknowledged that hedgehog signaling pathway plays crucial roles in cell proliferation, cell fate determination and cell differentiation; and its abnormal activation contributes to tumor development and progression [18–20]. It is documented that Sufu is a downstream negative regulator of Hh signaling pathway [36]. Sufu has been reported to serve as a tumor suppressor in pancreatic cancer [22], bladder cancer [24], glioma [37] and rhabdomyosarcoma [38]. With a view to clarify the potential molecular mechanisms by which LIFR-AS1 promotes breast cancer cell proliferation, migration and invasion, bioinformatics analyses and mechanistic investigations were performed. Moreover, mechanistic studies revealed that LIFR-AS1 interacts with miR-197-3p and that miR-197-3p mediates the effects of LIFR-AS1 on breast cancer cells.

RETRACTED

In sum, LIFR-AS1 is significantly down-regulated in both breast cancer tissues and cell lines, and exerts tumor-suppressing functions in breast cancer through miR-197-3p/Sufu axis. Our study may provide a basis for LIFR-AS1 as a candidate therapeutic target in breast cancer treatment. Hence, LIFR-AS1 may be used as a novel diagnostic biomarker and a promising therapeutic target for breast cancer.

## Abbreviations

FBS: Fetal bovine serum
Hh: Hedgehog
HRP: Horseradish peroxidase
LIFR-AS1: Leukemia inhibitory factor receptor antisense RNA 1
lncRNA: Long non-coding RNA
PBS: Phosphate-buffered saline
PBST: PBS containing 0.1% Tween-20
qRT-PCR: Quantitative real-time polymerase chain reaction
RIP: RNA-binding protein immunoprecipitation
Sufu: Suppressor of fused
TCGA: The Cancer Genome Atlas
